RETRACTED

# Blockage of transdifferentiation from fibroblast to myofibroblast in experimental ovarian cancer models

**DOI:** 10.1186/1476-4598-8-78

**Published:** 2009-09-27

**Authors:** Qin Yao, Xun Qu, Qifeng Yang, David A Good, Shuzhen Dai, Beihua Kong, Ming Q Wei

**Affiliations:** 1 Division of Molecular and Gene Therapies, Griffith Institute for Health and Medical Research, School of Medical Science, Griffith University, Gold Coast campus, Southport, Qld 4222, Australia; 2 Department of Obstetrics and Gynaecology, Qilu Hospital, Shandong University, Ji'nan 250012, Shandong, PR China; 3 Department of Obstetrics and Gynaecology, Affiliated Hospital of Qingdao University, Qing'dao 266003, Shandong, PR China; 4 Institute of Basic Medical Sciences, Qilu Hospital, Shandong University, Ji'nan 250012, Shandong, PR China

## Abstract

**Background:**

Tumour stromal myofibroblasts can promote tumour invasion. As these cells are genetically more stable than cancer cells, there has been enormous interest in developing targeted molecular therapies against them. Chloride intracellular channel 4 (CLIC4) and reactive oxygen species (ROS) have been linked with promoting stromal cell transdifferentiation in various cancers, but little is known of their roles in ovarian cancer. In this study, we examined the functional roles that both CLIC4 and ROS play in the process of ovarian cancer cell-stimulated or TGF-β1 induced fibroblast-to-myofibroblast transdifferentiation. We also examine whether it is possible to reverse such a process, with the aim of developing novel therapies against ovarian cancer by targeting activated transdifferentiated myofibroblasts.

**Results:**

We demonstrate that TGF-β1 induced or CM^SKOV3 ^activate transdifferentiated myofibroblasts (fibroblasts). These fibroblasts mimic "reactive" stromal myofibroblasts and demonstrate significant up-regulation of CLIC4 expression and increased level of ROS production. Blocking the production of ROS with an antioxidant consequently reduces the expression of CLIC4, and is accompanied by disappearance of *α*-smooth-muscle actin (α-SMA), a myofibroblast marker, suggesting ROS acts as a signalling molecule that promotes and enhances CLIC4 activities in the myofibroblast transdifferentiaton process. Down-regulation of CLIC4 with a generic agent or specific siRNA both significantly reduces the expression of factors related to the phenotypes and functions of myofibroblasts, such as α-SMA, hepatocyte growth factor (HGF) and vascular endothelial growth factor (VEGF), thus reversing the myofibroblast phenotype back to fibroblasts. These results convincingly show that ROS and CLIC4 are responsible for TGF-β1 induced fibroblast-to-myofibroblast transdifferentiaton and down-regulation of both is sufficient to block transdifferentiated myofibroblasts.

RETRACTED

**Conclusion:**

Molecular targeting of ROS and CLIC4 has the potential to develop novel therapies for ovarian cancer.

## Background

Ovarian cancer is not only common (1 in 67 women), but also is the most lethal gynaecological disease. It has, for years, been dubbed as a "silent killer" -- causing vague and non-specific symptoms until it is too advanced at the time of diagnosis [1]. Thus, ovarian cancer causes more deaths than any other type of gynaecological malignancies [1-3]. Even with the advent of modern treatments such as optimal cytoreductive surgery and systemic combination of chemotherapies, the 5-year survival rate for patients with advanced ovarian cancer has improved little; it is currently at as low as 10 - 30% [3].

Extensive studies have shed some lights on the complexity of ovarian cancer, and increasing evidence indicates that the disease development and progression are facilitated by interactions between tumour cells and activated stromal cells [4]. The tumour stroma (also referred to as "reactive stroma") is characterized by marked alterations in the phenotype and expression profile of "fibroblast-like cells". These cells commonly express *α*-smooth-muscle actin (α-SMA) and thus are termed as myofibroblasts [5,6]. Stromal fibroblasts are located at the tumour border near the invasion front. When these cells are activated by the tumour, they have a more profound influence on the development and progression of carcinomas than was previously appreciated [7]. Recent studies on reactive stroma in human breast carcinomas and in prostate cancer subjects have demonstrated that the co-culturing of myofibroblasts with these tumour cells can promote tumour invasion and angiogenesis [8,9]. Using an *in vitro *tumour-stroma model of skin carcinogenesis, Cat and colleagues (2006) demonstrated that myofibroblasts are recruited into cancer from different sources during cancer development and the invasion progression [10,11]. These cells were differentiated from the fibroblast population within the epithelial stroma after stimulation by transforming growth factor-β1 (TGF-β1) secreted by tumour cells. Tumour-associated myofibroblasts could also be transdifferentiated from non-malignant or epithelial derived carcinoma cells via epithelial-mesenchymal transition [11]. In addition, myofibroblasts could be recruited or derived from distant fibroblasts and bone marrow progenitor cells [12,13]. Although it has been shown that the conversion from fibroblasts to myofibroblasts constitutes the major source of myofibroblasts in tumour stroma, the molecular mechanisms underlying fibroblast-to-myofibroblast transdifferentiation is still not fully understood. Many questions remain, including what molecules are involved in the process and what roles are they playing?

RETRACTED

A family of intracellular chloride channels comprises seven highly homologous members (CLIC1-7). Recently, it was reported that one of them, the chloride intracellular channel 4 (CLIC4), a chloride channel of intracellular organelles, regulates intracellular pH and cell volume. Besides its presence on the organelle membrane, CLIC4 exists in soluble form in the cytoplasm and nucleus acting as a signalling protein or channel regulator [14]. The transcriptional level of CLIC4 is up-regulated when fibroblasts are induced by TGF-β1 and transdifferentiated into myofibroblasts, and more importantly CLIC4 is highly expressed in myofibroblasts of breast cancers [15]. Results from Littler and colleagues [16] shows that functional activity of CLIC4 depends on its redox state and that oxidative conditions enhance membrane binding and channel activity of CLIC4. More recent findings also reveal that reactive oxygen species (ROS) can alter the level of gene expression associated with cell differentiation, including fibroblast-to-myofibroblast transdifferentiation and epithelial-mesenchymal transition in liver fibrosis and some cancers [10,17,18]. However, the role of ROS in ovarian cancer and its relationship to CLIC4 in fibroblast-to-myofibroblast transdifferentiation process is not well understood. We hypothesized that the factors involved in fibroblast-to-myofibroblast transdifferentiation, such as tumour-cell-derived TGF-β1, promote the generation of intercellular ROS, which in turn acts as a signalling molecule, and initiates up-regulation of CLIC4 expression, thus triggering fibroblast-to-myofibroblast conversion. Agents that block ROS and CLIC4 might inhibit such transdifferentiation, which may delay myofibroblast-dependent tumour progression. Understanding these molecular interactions may assist with the development of novel molecular targeted therapies for ovarian cancer.

To test the hypothesis, we designed an experiment modelling ovarian cancer fibroblast-to-myofibroblast transdifferentiation and examined the pathway in which ROS and CLIC4 participates in fibroblast-to-myofibroblast transition induced by TGF-β1 or conditioned media from ovarian cancer SKOV3 cells (CM^SKOV3^). Furthermore, special agents were employed to down-regulate the production of ROS and CLIC4 in transdifferentiated myofibroblasts and such effects were assessed.

## Results and Discussion

### Myofibroblasts in the experimental ovarian cancer stroma have increased CLIC4 expression

Recent studies demonstrated that CLIC4 was markedly up-regulated in serum- or TGF-β1-stimulated fibroblasts isolated from breast cancer. These fibroblasts have a gene expression profile similar to myofibroblasts [15,19]. *In vivo*, the level of CLIC4 expression in the normal ovarian stroma is very low, but is significantly increased in the stroma of breast, kidney, oesophagus and colon cancers [20-22]. We hypothesised that CLIC4 may also play an important functional role in causing stromal fibroblast to myofibroblast transdifferentiation, which is critical in ovarian cancer development and progression.

RETRACTED

Ovarian surface epithelium is in fact a single layer of mesothelial cells covering the ovarian surface and contiguous with coelomic mesothelium. We recently showed that the expression of CLIC4 was readily detected in epithelia and stroma of these primary epithelial ovarian cancers in 96.7% (29/30) of patients. Moreover, the expression of CLIC4 in cancer stroma was correlated with up-regulation of a well-accepted myofibroblast marker, α-SMA, which was detected in 93.3% (28/30) of the same stroma (Yao et al., manuscript in preparation).

In order to define the expression of CLIC4 in transdifferenciated myofibroblasts we performed immunohistochemical staining of CLIC4 and α-SMA1 (Fig. 1A). We used a myofibroblast conversion culture model where ovarian primary fibroblasts and/or human fibroblast MRC-5 cells were co-cultured with CM^SKOV3 ^or TGF-β1. Fig. 1A showed that the myofibroblasts displayed a significant increase in CLIC4 expression both in the cytoplasm and nucleus (p < 0.05) with co-expression of a myofibroblast marker, α-SMA in the cytoplasm in the presence of CM^SKOV3 ^or 10 ng/ml TGF-β1 compared with the serum-free medium control (p < 0.05). Furthermore, the immunoblot and real time qRT-PCR data provides strong evidence that the increased amounts of α-SMA and CLIC4 expression in myofibroblasts were up-regulated both at the transcription and protein levels (*P *< 0.05) (Fig. 1B). These results confirmed that the expression of CLIC4 was up-regulated during fibroblast to myofibroblast conversion when induced by TGF-β1 or activated by CM^SKOV3 ^suggesting that CLIC4 directly participates in stromal fibroblast activation in ovarian cancer.

**Figure 1:** **Immunohistochemical staining of CLIC4 and α-SMA**. (A). In cultured fibroblasts (control) and transdifferiated myofibroblasts (activated by CM^SKOV3 ^(CM) and TGF-β1). Scale bar, 50 μm. (B) Western blot of MRC-5 cells or primary ovarian fibroblasts cultured in serum-free medium (control), in CM or TGF-β1 for 48 hours.

### ROS mediates up-regulation of CLIC4, which leads to myofibroblast transdifferentiation

More recent reports have suggested that ROS acts as a signalling molecule of TGF-β1 in the regulation of myofibroblast differentiation in liver fibrosis and an *in vitro *tumour-stroma model of skin carcinogenesis [10,17]. It can alter gene expression levels by regulating the expression of multiple phenotypic markers, such as α-SMA [10]. When we examined the intracellular ROS levels in MRC-5 fibroblasts treated with 10 ng/ml TGF-β1 or CM^SKOV3^, we showed a significant increase in the fluorescence intensity using DCF-DA dye staining, indicating high levels of intracellular ROS production (Fig. 2A). Simultaneously, the high level of ROS was accompanied by up-regulation of α-SMA and CLIC4 expressions in the myofibroblasts. However, when the MRC-5 fibroblasts cells were pre-treated with the antioxidant N-acetylcysteine (NAC), which blocked the intracellular ROS, the up-regulation of α-SMA and CLIC4 expressions, stimulated by TGF-β1 or CM^SKOV3^, were also reduced at both mRNA and protein levels (Fig. 2C). These results showed that not only α-SMA but also CLIC4 transcription and translation levels were significantly up-regulated followed by generation of ROS during TGF-β1 induced fibroblast-to-myofibroblast differentiation. This effect could be blocked by treatment with the NAC. This is the first evidence that showed TGF-β1 or CM^SKOV3 ^stimulated the production of cellular ROS and CLIC4, which correlated with myofibroblast transdifferentiation (Figure 2). Moreover, agents which inhibit ROS alleviated the expression of CLIC4 and α-SMA.

RETRACTED

**Figure 2:** **ROS-mediated up-regulation of CLIC4 expression during myofibroblast transdifferentiation**. (A) CM^SKOV3 ^and TGF-β1 induced oxidative stress in MRC-5 fibroblasts using DCF-DA analysed by fluorescent microscopy. Scale bar, 50 μm. (B, C), Myofibroblast transdifferentiation was dependent on ROS. The expression of α-SMA and CLIC4 was determined by real time RT-PCR and Western blot, using MRC-5 cells treated with or without 5 mM of antioxidant (NAC), before addition of CM^SKOV3 ^and TGF-β1. * *P *< 0.05. (D), ROS mediated up-regulation of CLIC4 expression in both cytoplasm and nucleus during myofibroblast transdifferentiation. CLIC4 protein expression in cytoplasm and nucleus was determined by Western blot analysis. Fibroblasts cultured in serum-free medium served as control for all the experiments.

CLIC4 shares homology with that of the glutathione S-transferase (GST) superfamily, suggesting its function may depend on the cellular redox state. A cysteine at position 35 preceding the N-terminal transmembrane domain is redox sensitive and is modified by glutathione [16]. CLIC4 subcellular locations are critical in its physiological functions [23]. Since CLIC4 is upregulated in myofibroblasts, we further assessed the expression of CLIC4 in the nucleus and cytoplasm during myofibroblast differentiation using Western blot. As shown in Fig. 2D, the expression of CLIC4 increased not only in the cytoplasm but also in the nucleus, particularly when fibroblasts were treated with TGF-β1 or CM^SKOV3^. Pre-treatment with antioxidant NAC also reduced both cytoplasmic and nuclear CLIC4 expressions. Taken together, these data suggest that TGF-β1 or CM^SKOV3 ^increases cellular ROS, which induces up-regulation and activity of CLIC4, leading to myofibroblast transdifferentiation.

RETRACTED

### Down-regulation of CLIC4 reverses the myofibroblast phenotype

A previous study reported that up-regulation and nuclear translocation of CLIC4 was responsible for expression of keratinocytic differentiation markers by altering chloride content and pH of the nucleus. Treatment of keratinocytes with a chloride channel inhibitor blocked the chloride ion flux by nuclear-specific CLIC4 and reduced the expression level of differentiation biomarker K10 [21]. In addition to the channel activity of CLIC4, there was a report that showed CLIC4 could promote cytoskeleton function by interaction with dynamin, tubulin, actin and 14-33 proteins [24]. Recombinant CLIC4 was shown to reduce cell motility in fibroblasts [15]. Thus, the relationship between CLIC4 and α-SMA seems to be important to the physiological function of myofibroblast cells. Since CLIC4 is the only intracellular chloride channel that can be induced by TGF-β1 in fibroblasts [15], we used a chloride channel inhibitor, indanyloxyacetic acid 94 (IAA-94) to inhibit the function of CLIC4 and found reduced expression of α-SMA and myofibroblast-mediated angiogenesis factors. Using a CLIC4 specific siRNA, we further demonstrated the consequential outcome of reduced CLIC4 expression. When fibroblasts were transfected with specific CLIC4 siRNA prior to treatment with TGF-β1 or CM^SKOV3 ^CLIC4, siRNA efficiently down-regulated CLIC4 transcript levels by an average of 90%. The induction of α-SMA transcript induced by TGF-β1 or CM^SKOV3 ^was significantly blocked in CLIC4 siRNA-transfected fibroblasts (Fig. 3A, B). At the protein level, immunoblot and immunofluorescent data showed that silencing of CLIC4 prevented the expression of α-SMA (Fig. 3C, D). These results are in agreement with those of a previous study by Suh *et al.*, who have reported that α-SMA protein level in fibroblasts increases significantly upon CLIC4 over expression produced by infecting with recombinant CLIC4 adenovirus [20]. Additionally, we found that silencing CLIC4 reversed the up-regulation of angiogenic factors, ie.: hepatocyte growth factor (HGF) and vascular endothelial growth factor (VEGF) in TGF-β1 or CM^SKOV3 ^treated fibroblasts (Fig. 3E, F, G).

RETRACTED

**Figure 3:** **Specific inhibition of CLIC4 expression stops myofibroblast transdifferentiation to fibroblast**. MRC-5 cells were transfected with specific CLIC4 siRNA and then treated with or without CM^SKOV3 ^and TGF-β1. Mock transfection with transfection reagent alone and scrambled siRNA (neg siRNA) served as negative controls. The relative levels of CLIC4 (A), α-SMA (B) transcripts and α-SMA protein expression were assessed by real time RT-PCR, Western blot (C) and immunofluorescent staining (D). Scale bar, 50 μm. Quantitative RT-PCR was used to analyse transcription levels of pro-angiogenic factors, VEGF (E), HGF (F) and α-SMA (G) in MRC-5 cells treated with chloride channel inhibitor IAA-94, NAC or CLIC4 siRNA before addition of CM^SKOV3 ^and TGF-β1. * *P *< 0.05.

Angiogenesis plays a key role in tumour development by supplying the tumour with oxygen and nutrients. Recent data shows that myofibroblasts are the major cell type expressing pro-angiogenic factors in cancer stroma such as angiogenic factor VEGF [12]. In this study EGF CM^SKOV3 ^or TGF-β1 activated myofibroblasts have higher levels of expressions of HGF and VEGF when compared to inactivated fibroblasts (Fig. 3). Pre-treatment with a chloride channel inhibitor IAA-94 to block function of CLIC4 lowered HGF and VEGF expression levels in myofibroblasts by 24% - 80%. Furthermore, after fibroblasts were relieved from these treatments, exposure to CM^SKOV3 ^or TGF-β1 restored the expression of factors related to the phenotype and functions of myofibroblasts (data not shown), indicating these repressing activities were due to the activation by CM^SKOV3 ^or TGF-β1, and were not mere cytotoxic effects.

## Conclusion

Ovarian cancer, like most solid tumours, not only acquires adaptive mutations during therapy, but interacts with myofibroblasts, thus promoting further growth and metastasis. Because myofibroblasts are genetically more stable than cancer cells, therapeutic targeting of these myofibroblasts in the stroma has distinct advantage and potential. In this study, we showed that treatment of myofibroblasts with agents blocking ROS or CLIC4 can reverse the phenotype of myofibroblasts, and markedly repress the production of angiogenesis factors associated with myofibroblast transdifferentiation, indicating that ROS or CLIC4 are excellent targets for the development of targeted molecular therapies for the treatment of ovarian cancer.

## Materials and methods

### Cell culture and in vitro culture models

Both human epithelial ovarian cancer cell line SKOV3 and human foetal lung fibroblast cell line MRC-5 were obtained from Basic Medicine Research Institute, Qilu Hospital, Shandong University, P.R. China. Human ovarian primary fibroblasts were isolated as described previously [25]. These cells were cultured in DMEM (Gibco) containing 10% heat-inactivated foetal bovine serum (Gibco) and 100 units/ml penicillin/streptomycin. The cultures were maintained at 37°C in an atmosphere of 5% CO_2_. The purity of primary stromal cells was more than 98% confirmed by keratin and vimentin staining [26]. Ovarian fibroblasts between passage 3 and 8 were used for all experiments.

RETRACTED

### Treatment of cells with TGF-β1, conditioned medium from SKOV3 (CM^SKOV3^), N-acetyl-L-cysteine (NAC) or IAA-94

After SKOV3 cells were cultured in serum-free medium for 48 h, the conditioned medium were collected, clarified by centrifugation and stored at -20°C for future use.

When MRC-5 cells and human ovarian primary fibroblasts reached subconfluence, the medium was replaced by serum-free medium, serum-free medium with 10 ng/ml human recombinant TGF-β1 (PeproTech EC Ltd., UK) or CM^SKOV3^, then cultured for another 48 hours. In order to study the inhibitory functions of NAC and IAA-94, subconfluent fibroblasts were incubated with 5 mM NAC for 4 hours or 10 μM IAA-94 for 24 hours before addition of TGF-β1 or CM^SKOV3^.

### Immunochemical and immunofluorescent staining

For immunohistochemical staining, the sections were deparaffinized, and rehydrated followed by antigen retrieval. The cells were fixed with 3.7% formaldehyde for immunocytochemical analysis. Afterwards, these sections and cells were blocked with 10% normal goat serum, and then incubated with rabbit anti-CLIC4 polyclonal antibody (Lifespan Biosciences, USA) and rabbit anti-α-SMA monoclonal antibody (Abcam, UK) at 4°C overnight, respectively. After washing with PBS, the slides were incubated with anti-rabbit IgG secondary antibody for 45 min and then incubated with biotinylated horseradish peroxidase solution for 45 min. Finally, the slides were stained with diaminobenzidine and observed under light microscope. For immunofluorescent staining, cells were stained with FITC conjugated anti-rabbit IgG secondary antibody, and nuclei were stained with 4,6-diamidino-2-phenylindole (DAPI). Images were recorded using confocal microscope.

### Western blot analysis

Cells were lysed in RIPA lysis buffer plus protease inhibitors. Cell nuclear and cytoplasmic proteins were extracted using Nuclear/Cytosol Extraction Kit (Pierce Biotechnology, Inc., USA). The expressions of CLIC4 and α-SMA were characterized by Western blot using polyclonal anti-CLIC4 antibody and monoclonal anti-α-SMA antibody as primary antibodies. Reaction products of β-actin were used to normalize the intensities between lanes.

RETRACTED

### Analysis of intracellular ROS

The intracellular ROS generation was assayed using 2'-7'-dichlorofluorescein diacetate (DCF-DA) (Sigma) dye as previously described [10].

### Small interfering RNA (siRNA) transfection

The siRNAs used in this study were designed, functional tested by and purchased from Qiagen. The sequences of siRNA were as follows: CLIC4 validated siRNA 5'-GCAGUACAAUGAU UAGUAAdTdT-3' (sense) and 5'-UUACUAAUCAUUGUACUGCdTdA-3' (antisense); negative Control siRNA 5'-UUCUCCGAACGUGUCACGUdTdT-3' (sense) and 5'-ACGUGACACGU UCGGAGAAdTdT-3' (antisense); MAPK1 positive control siRNA 5'-UGCUGACUCCAAA GCUCUGdTdT-3' (sense) and 5'-CAGAGCUUUGGAGUCAGCAdTdT-3' (antisense). Lipofectamine 2000 reagent was used for transfection with a final concentration of 30 nM of each siRNA. After 16 hours of incubation of transfection, cells were replaced with serum-free medium with or without 10 ng/ml TGF-β1 or CM^SKOV3 ^and then incubated for another 48 hours.

### Real-time Quantative Polymerase Chain Reaction

Total RNA was extracted from cells using Trizol reagent (Invitrogen). RNA was reverse transcribed with oligo (dT) and M-MLV reverse transcriptase (Promega). The primers were designed as follows: α-SMA (accession no. NM_001613), 5'-AGGTAACGAGTCAGAGCTTTGGC-3' (forward) and 5'-CTCTCTGTCCACCTTCCAGCAG-3' (reverse); CLIC4 (accession no. NM_013943), 5'-CACGTAAATTTCTGGATGGCAATG-3' (forward) and 5'-ATCACTGGGACAGGTATTGGTGAAC-3' (reverse); VEGF (accession no. NM_001025366), 5'-CCTGGTGGACATCTTCCAGGAGTACC-3' (forward) and 5'-GAAGCT CATCTCTCCTATGTGCTGGC-3' (reverse); HGF (accession no. NM_000601), 5'-GTAAATG GGATTCCAACACGAACAA-3' (forward) and 5'-TGTCGTGCAGTAACAACCAACTC-3' (reverse); β-actin (accession no. NM_001101), 5'-AACTCCATCATGAAGTGTGA-3' (forward) and 5'-ACTCCTGCTTGCTGATCCAC-3' (reverse). β-actin was chosen as the house keeping gene. The quantification was performed using SYBR Green (Takara Biotechnology, Inc., Japan). Samples were analysed using LightCycler^® ^2.0 Instrument (Roche Applied Science, Switzerland).

### Statistical analysis

The data represented means ± S.D. of three independent experiments. Statistical differences were analysed with the Student's *t*-test. Differences were considered significant at *P*-values < 0.05.

## List of abbreviations

CLIC4: chloride intracellular channel 4; DCF-DA: 2'-7'-dihydrodichlorofluorescein diacetate; NAC: N-acetyl-L-cysteine; ROS: reactive oxygen species; siRNA: small interfering RNA; TGF-β1: transforming growth factor-β1

RETRACTED

## Competing interests

The authors declare that they have no competing interests.

## Authors' contributions

QY - day to day bench researcher, generated most of the data, and drafted the manuscript; XQ - initial help to QY on cell culture, immunoblots; QfY - initial help to QY on cell culture, immunblots, and Western blots; DAG - revised the paper and created some figure; SD - initial supervision of Q Y, provided help with interpreting data. BK - initial supervision of QY, provided help with interpreting data. MQW - head of the laboratory, initiated the collaboration, supervised QY on day to day bench work, analysed the data and wrote the manuscript. All authors read and approved the final manuscript.

## Authors' information

QY is a visiting fellow (supported by MW) to Professor Ming Wei's laboratory at the Division of Molecular and Gene Therapies, Griffith University at Gold Coast campus.
